The article "IL-6 Promotes Cancer Stemness and Oncogenicity in U2OS and MG-63 Osteosarcoma Cells by Upregulating the OPN-STAT3 Pathway" was retracted in 2021. Reason: duplicated images.

# IL-6 Promotes Cancer Stemness and Oncogenicity in U2OS and MG-63 Osteosarcoma Cells by Upregulating the OPN-STAT3 Pathway

**DOI:** 10.7150/jca.29931

**Published:** 2019-10-21

**Authors:** Chuan Zhang, Kun Ma, Wu-Yin Li

**Affiliations:** Luoyang Orthopaedic-Traumatological Hospital and Henan Orthopaedic Hospital, Luoyang, Henan 471002, China.

**Keywords:** IL-6, osteosarcoma, stemness, chemoresistance, invasion, migration, osteopontin, STAT3

## Abstract

**Background:** Cancer stem cells (CSCs) are associated with tumor development, chemoresistance, recurrence, metastasis, and even prognosis. Interleukin (IL)-6 overexpression has been implicated in the development of various cancers, including osteosarcoma. This study aimed to investigate the role of IL-6 in modulating clinicopathological features, malignant traits, and stemness in osteosarcoma, and to determine the mechanisms underlying IL-6-mediated osteosarcoma progression. **Methods:** Patients with osteosarcoma (n = 54) and healthy controls (n = 50) were selected. No patients received any pre-operative cancer treatment. Serum levels of IL-6 were determined in patients with osteosarcoma by ELISA and their relationship with pathological features and prognosis analyzed. The 3-(4,5-dimethyl -2-thiazolyl)- 2,5-diphenyl-2H-tetrazolium bromide (MTT) and colony formation assays were used to evaluate cell proliferation, transwell assays were used to assess the invasive potential of cells, and cell migration rates were analyzed using a wound healing assay. Tumor self-renewal was detected using a spheroid formation assay and CD133 and CD44 expression assessed by flow cytometry. Protein levels of NANOG, SOX2, OCT3/4, OPN, and epithelial-to-mesenchymal transition (EMT)-related markers, and the phosphorylation status of STAT3, were determined by western blotting. Finally, cell viability was determined with or without cisplatin (cis-dichlorodiammineplatinum [DDP])/adriamycin (ADR) treatment. Xenograft tumor models were established by subcutaneous injection of osteosarcoma spheroids, with or without IL-6. **Results:** Serum IL-6 levels were higher in osteosarcoma patients than controls. There was no significant association of serum IL-6 level with age, sex and tumor size; however, it was associated with TNM stage, and lung metastasis (P < 0. 05). IL-6 significantly increased proliferation and colony formation of osteosarcoma cells, and enhanced their invasion and migratory potential, thus promoting an EMT-like phenotype and elevated chemoresistance of to DDP/ADR. Spheroid size/proportion of CD133^+^CD44^+^ cells and SOX2, OCT3/4, and NANOG protein levels were elevated by IL-6 treatment in a time-dependent manner; however, IL-6 did not substantially influence any of these features in hFOB 1.19 and T98G cells. Knockdown of IL-6 reduced cell viability, colony formation, and invasion/migration ability, and reversed EMT, whereas it increased chemosensitivity to DDP/ADR. Blocking IL-6 expression with siRNA also caused loss of stemness, including reducing self-renewal ability, and reduced the proportion of CD133/CD44-positive cells, and expression of stemness-related genes. Pretreatment with the STAT3 inhibitor, S3I-201, decreased sphere size, and downregulated NANOG, SOX2, and OCT3/4 protein levels, compared with IL-6 treatment alone. Furthermore, OPN levels were elevated in response to IL-6 and an anti-OPN antibody effectively blocked IL-6-induced spheroid formation and STAT3 phosphorylation. *In vivo*, tumor size and weight were higher in IL-6 treated mice than controls. **Conclusions:** IL-6 mediates promotion of osteosarcoma spheroid stemness by activating OPN/STAT3 signaling.

## Introduction

Osteosarcoma is characterized by spindle stromal cells that create new bone tissue, and is one of the most common malignant bone tumors worldwide, occurring primarily in children and adolescents 1. A combination of surgery with adjuvant chemotherapy 2, using cisplatin (cis-dichlorodiammineplatinum, DDP) and adriamycin (ADR), has been proposed as a means to improve the 5-year survival rate of patients with osteosarcoma; nevertheless, overall survival remains low for patients with osteosarcoma, and disease recurrence and primary or secondary chemoresistance are the leading causes of poor clinical outcomes 3. Cancer stem cells (CSCs), as defined by the American Association for Cancer Research, are small subpopulations of cells with properties of self-renewal, differentiation, increased rates of tumorigenesis, and sustained tumor growth, which cause chemoresistance and disease recurrence, and lead to cellular invasion and migration. Traditional cancer therapies can reduce the size of primary tumors, but do not affect CSCs^4^; therefore, the development of CSC-targeted therapies has the potential to prevent tumor recurrence and increase the survival rate of patients with osteosarcoma.

The tumor microenvironment, which contains stromal cells, immune cells, cytokines, growth factors, and hypoxic factors, can control the aggressiveness of many tumor types 5-6. Interleukin-6 (IL-6) is produced and secreted by various cell types, including tumor cells, is a pro-inflammatory molecule, whose overexpression has been reported in serum and tumor samples from patients with various types of cancer, including prostate cancer 7, multiple myeloma 8, renal cell carcinoma 9, and breast cancer 10. Upregulation of IL-6 is positively associated with high rates of tumor growth and poor therapeutic response 7. In addition, IL-6 promotes the stemness of lung 11, breast 12, and colon 13 cancer cells, among others.

Osteopontin (OPN) is a secreted phosphorylated glycoprotein, which interacts with cells through various integrin molecules, including a4b1, a9b1, a9b4, av (b1, b3, b5), and CD44 14. Elevated OPN levels contribute to enhanced chemoresistance and increased osteosarcoma migration 15. OPN expression was also identified as a biomarker associated with increased risk of developing osteosarcoma 16. Further, Wang et al demonstrated that IL-6 enhances cancer stemness and promotes the migration of hepatocellular carcinoma cells via upregulation of OPN 17; however, there have been no reports of studies to determine which effects of OPN can modulate the malignant traits of osteosarcoma.

Serum levels of IL-6 are significantly higher in patients with osteosarcoma than those in healthy individuals 18-19. Endogenous IL-6/IL-6-related signaling contribute to elevated proliferation/ chemoresistance of osteosarcoma cells, and induce their epithelial-to-mesenchymal transition (EMT), thus promoting their migration and invasion 20. Furthermore, Han et al. reported that osteosarcoma cells become more sensitive to cisplatin when IL-6 production is reduced 21; however, little is known about the relationship between IL-6 expression and the clinicopathological characteristics of patients with osteosarcoma. Moreover, there are no data indicating whether IL-6 can modulate the malignant traits of osteosarcoma, including maintenance/promotion of stemness. In the present research, we explored the role of IL-6 in regulation of osteosarcoma stemness, as well as the underlying mechanisms, to provide experimental evidence to support therapeutic targeting of IL-6.

## Materials and methods

### Patients and clinical specimens

Patients with osteosarcoma (n = 54) and healthy controls (n = 50) were selected. None of the patients received any preoperative cancer treatment. Clinical samples were collected from patients after obtaining informed consent, approved by the Luoyang Orthopedic Hospital and Orthopedic Hospital of Henan (Luoyang, China). Serum IL-6 levels in patients with osteosarcoma were detected by enzyme-linked immunosorbent assay (ELISA) and their relationship with the pathological features and prognosis analyzed.

### Reagents

U2OS and MG-63 osteosarcoma cells and *hu*man normal osteoblastic hFOB 1.19 cells were obtained from the Shanghai Institute of Biochemistry and Cell Biology (Chinese Academy of Sciences, Shanghai, China). The human glioblastoma cell line, T98G, was purchased from American Type Culture Collection (Rockville, MD, USA). Dulbecco's Modified Eagle Medium (DMEM) cell culture medium and fetal bovine serum (FBS) were purchased from Hangzhou Sijiqing Biological Engineering Material Co. Ltd. (Hangzhou, Zhejiang, China). Antibodies against OPN were purchased from Abcam (Cambridge, MA). N-acetyl cysteine and recombinant human IL-6 were purchased from Sigma (St. Louis, MO, USA). Enhanced chemiluminescence (ECL) western blotting kits were obtained from Santa Cruz Biotechnology, Inc. (Santa Cruz, CA, USA).

### Cell culture

U2OS, MG-63 cells, and T98G cells were grown in DMEM containing 10% FBS, 100 μg/ml penicillin, and 100 μg/ml streptomycin at 37°C in a 5% CO2 incubator. The human normal osteoblastic cell line, hFOB 1.19, was maintained in DMEM/F-12 (Gibco) supplemented with 10% FBS (Gibco) and 0.3 mg/mL geneticin (G418; Gibco) at 37°C in a humidified atmosphere containing 5% CO2.

### Sphere formation assay

To enrichment for spheroids, cells were isolated, reseeded in ultralow attachment 96-well plates (Corning Inc., Life Sciences), and cultured in DMEM/F-12 (Invitrogen) serum-free medium containing B27 (Invitrogen), containing 20 ng/ml epidermal growth factor (Peprotech, Rocky Hill, NJ, USA), 20 ng/ml basic fibroblast growth factor (Peprotech), 10 ng/ml hepatocyte growth factor (Peprotech), and 1% methylcellulose (Sigma), for 10 days. Spheres were then counted by inverse microscopy and cell colonies with a diameter > 50 µm measured. In subsequent experiments, cells were treated with 50 ng/ml IL-6.

### Colony formation assay

hFOB 1.19, U2OS, MG-63, and T98G cells were seeded at a density of 250 cells/well in 24-well plates, treated with 50 ng/ml IL-6 for 24, 48, and 72 h, then stained with 1% methylrosanilinium chloride, and the numbers of visible colonies counted. Relative colony formation ability was calculated as follows: Relative colony formation ability = (mean experimental colony number/mean control colony number) x 100%.

### Morphological observation

An Olympus phase-contrast microscope was used to observed the cell morphology of hFOB1.19 cells which were seeded in six-well plates at the density of 1 × 105 cells/well. The cells were then treated with or without IL-6 for 24 h,48 h, 72 h. Cell morphology was observed through phase - contrast microscopy.

### Flow cytometry

U2OS and MG-63 cells were treated with 50 ng/ml IL-6 for 24, 48, and 72 h, then harvested and washed with 2% FBS/phosphate-buffered saline (PBS) solution, followed by incubation with antibodies against CD133 and CD44 (1:100) for 60 min. Cells were then washed and incubated with fluorescein isothiocyanate (FITC)-labeled secondary antibodies for 30 min. Next, cells were washed twice and resuspended in 100 μl fluorescence-activated cell sorting (FACS) buffer. Stained cells were then analyzed by flow cytometry (FACS Calibur, BD Bioscience, USA).

### Western blotting

Cells were washed in phosphate buffered saline (PBS) and resuspended at room temperature. After incubation on ice for 30 min, cells lysates were centrifuged at 14,0009 x g at 4°C. Protein concentrations were measured using Bradford protein assay reagent, with bovine serum albumin as a standard. Membranes were incubated overnight at 4°C with primary antibodies (all at 1:1000) against the following molecules: phosphorylated- (p-)STAT3 or caspase 3 (Abcam, Cambridge, MA, USA); STAT3, GAPDH, a-SMA, and E-cadherin, Vimentin, NANOG, OCT4, SOX2, or OPN (Cell Signaling Technology, Danvers, MA, USA). Membranes were then incubated with secondary antibodies (1:5000) at room temperature for 2 h. GAPDH was used as a loading control.

### Transwell assay

As described previously, cells were seeded in 10 mm diameter transwell plates, with 8-µm pore polycarbonate filters. The upper and lower compartments of the plates were separated by a filter coated with 25 mg of matrigel, which formed a reconstituted basement membrane at 37°C. After treatment with 50 µg/ml of IL-6 for 0, 24, 48, and 72 h, cells were seeded into the upper well, while the lower well was filled with DMEM containing 10% FCS. After incubation in the presence of 5% CO2, cells were fixed for 30 min in 4% formaldehyde and stained for 15 min. Non-migrating cells were then removed from the upper surface (inside) of the transwell with a wet cotton swab, and cells that had migrated or invaded the bottom surface of the filter counted. Six evenly spaced fields of cells were counted in each well using an inverted phase-contrast microscope.

### Wound healing assay

Cells were seeded in 6-well plates at a density of 5 × 10^5^ per well in DMEM supplemented with 10% FBS. Twelve hours after seeding, cells were treated with IL-6 (50 µM) or an equivalent volume of DMSO for 48 h. A scratch was then made in the cell monolayer, and the rate of wound closure observed at 24 and 48 h, and analyzed using Image J software.

### Tumor xenografts

Male BALB/c nude mice (6 weeks old, 18-20 g) were obtained from the Shanghai Experimental Center, Chinese Science Academy. All procedures followed the guidelines issued by the National Institute of Health, and this study was approved by the Animal Ethics Committee of Luoyang Orthopaedic-Traumatological Hospital (TCM-2015-018-E20). Cells (1 × 10^5^ per ml) were suspended in 100 μl of PBS (Hyclone) and Matrigel (BD Pharmingen) mixed (1:1), and implanted subcutaneously at the point where the left forelimb joins the trunk. The volume of the subcutaneous tumors was monitored every 3 days for 3 weeks. Tumors were measured using electronic calipers, and tumor volume estimated using the formula:Tumor volume = ½ x a × b^2^ where 'a' and 'b' are the longest and shortest diameters of the tumor, respectively. After 3 weeks, mice that had sizeable tumors (≥ 3 mm in diameter) were considered tumor-bearing. The number of tumor-bearing mice in each group was counted. Tumors were removed and soaked in 10% neutral-buffered formalin for paraffin embedding.

### Statistical analysis

Data are presented as means ± SD. Differences between groups were analyzed using the Student's t-test. Statistical analyses were performed using SPSS software version 16.0 (SPSS, Inc.). *P* < 0.05 was considered statistically significant.

## Results

### 1. IL-6 levels are associated with tumor progression and lung metastasis

In this study, we evaluated plasma IL-6 levels in 54 patients with osteosarcoma and 50 healthy individuals and assessed the relationship between IL-6 levels and patient clinicopathological features. Compared with the healthy control group, IL-6 expression was clearly elevated in patients with osteosarcoma (Fig. 1; Table 1). As shown in Table 2, levels of serum IL-6 expression were not associated with age ,sex and tumor size (P > 0.05), while they were associated with TNM stage, as well as lung metastasis (P < 0.05).

### 2. The effect of IL-6 on proliferation of osteosarcoma cells

To investigate the effect of IL-6 on the viability of MG-63/U2OS-derived CSCs, cells were treated with 50 μM IL-6 for 0-72 h and then subjected to 3-(4,5-dimethyl-2-thiazolyl)-2,5-diphenyl-2H-tetrazolium bromide (MTT) assays. As shown in Figure 2A, IL-6 clearly increased the proliferation of U2OS/MG-63 cells in a time-dependent manner (P < 0.05); however, it did not substantially influence hFOB 1.19 or T98G cell viability.

Additionally, colony formation assays showed that, compared with untreated cells, IL-6 significantly increased the clonogenicity of U2OS/MG-63 cells, in a dose-dependent manner (Fig. 2B, C), although it did not promote clonogenicity of hFOB 1.19 and T98G cells (P < 0.05). Significantly, as shown in Figure 2D and 2E, knockdown of IL-6 using siRNA led to reduced clonogenicity of U2OS/MG-63 cells compared with the si-control group (P < 0.05).

### 3. IL-6 accelerates osteosarcoma invasion and migration, and promotes EMT

The invasion and migration of tumor cells is a primary cause of mortality in patients with cancer. As shown in Figure 3A and B, transwell assays revealed that IL-6 treatment significantly promoted U2OS/MG-63 cell invasion, as numbers of invasive cells increased in a time-dependent manner (P < 0.05), consistent with previous studies 22-23. IL-6 also increased migration of osteosarcoma cells, leading to significantly lower wound widths in treated cells compared with controls over time (Fig. 3C, 3D). Meanwhile, the ability of hFOB 1.19 and T98G cells to invade/migrate was not significantly changed in response to IL-6 treatment (*P* < 0.05).

EMT is a dynamic biological process via which epithelial cells develop properties of mesenchymal cells. EMT of cancer cells ultimately leads their metastasis 24. Qu et al discovered that spheroid formation by osteosarcoma stem cells was suppressed when EMT was reversed 25. Similarly, our data show that Vimentin, a-SMA, and MMP-2 levels were upregulated, while those of E-cadherin were decreased in MG-63/U2OS cells in response to IL-6 (Fig. 3E, F). Consistent with these finding, IL-6 had no significant negative effects on expression of EMT-related markers in hFOB 1.19 and T98G cells (*P* < 0.05).

As shown in Figure 3G-J, MG-63/U2OS cells treated with si-IL-6 exhibited decreased invasiveness and significantly increased wound widths compared with the si-control group (P < 0.05). Consistent with the results presented above, si-IL-6 also attenuated expression levels of Vimentin, a-SMA, and MMP-2 and increased those of E-cadherin (Fig. 3K, L). Overall, these results demonstrate that IL-6 could elevate the invasion/migration abilities only of MG-63/U2OS cells (P < 0.05).

### 4. IL-6 promotes osteosarcoma chemoresistance

Previous studies have shown that downregulation of IL-6 can abrogate chemoresistance in colon and breast cancer 26-28. To assess whether IL-6 contributes to DDP/ADR- chemoresistance in U2OS/MG-63 cells, MTT analysis was used to assess the viability of MG-63/U2OS cells treated with DDP/ADR in the presence or absence of IL-6. As shown in Figure 4A and 4B, IL-6 increased the viability of U2OS and MG-63 cells in response to treatment with DDP/ADR, compared with the DDP/ADR alone group (P < 0.05), while there was no clear change detected in the viability of hFOB 1.19 and T98G cells treated in the same way. Consequently, as shown in Figure 4C and 4D, pretreatment of cells with si-IL-6 significantly attenuated the viability of U2OS and MG-63 cells in the presence of DDP/ADR (P < 0.05).

### 5. IL-6 promotes tumorigenesis and stemness in MG-63/U2OS derived CSCs

Sphere formation is regarded as a defining trait of CSCs 29. Compared with the control group, U2OS/MG-63 CSCs treated with IL-6 increased in number and sphere diameter (Figure 5A, B), consistent with the findings of previous studies. Remarkably, IL-6 failed to increase the size of T98G CSCs. Also,the morphological changes of hFOB1.19 cells were not been observed(P<0.05). CD133-positive subpopulations of SAOS2, MG63, and U2OS osteosarcoma cells exhibit stem-like properties 30. CD44 is a type I transmembrane glycoprotein that mediates cell-cell and cell-matrix interactions through its affinity for hyaluronic acid 31. As shown in Figure 5C-F, levels of CD133 and CD44 were simultaneously upregulated in response to treatment with IL-6, compared with the control group. The numbers of CD133-and CD44-positive cells appeared to plateau at 72 h (*P* < 0.05).

NANOG, SOX2, and OCT3/4 are key factors in maintaining the pluripotency of osteosarcoma CSCs. Consistent with the results of flow cytometry, the data in Figure 5G demonstrate that protein levels of NANOG, SOX2, and OCT3/4 were simultaneously upregulated in U2OS/MG-63 CSCs in response to IL-6, peaking at 72 h. Furthermore, the expression of NANOG, SOX2, and OCT3/4 in T98G CSCs did not change significantly following IL-6 treatment.

Additionally, the sizes of tumor spheres, as well as OCT4, SOX2, and NANOG levels, were significantly suppressed in cells treated with si-IL-6 compared with the si-control group (P < 0.05). We conclude that IL-6 can confer stemness on U2OS/MG-63 CSCs.

### 6. STAT3 signaling promotes IL-6-mediated stemness in osteosarcoma cells

Aberrant STAT3 pathway activation is a mechanism that contributes to CSC maintenance 32. Honoki et al. showed that MG-63-derived CSCs had elevated mRNA expression levels of stem cell-related genes, as well as STAT3 33, and activation of STAT3 is involved in osteosarcoma cell survival and drug resistance. As shown in Figure 6A and 6B, STAT3 phosphorylation was increased in response to IL-6. Based on these data, combined with the results presented above, we theorized that the STAT3 pathway may participate in IL-6-mediated U2OS/MG-63 cell cytotoxicity. To test this hypothesis, we conducted further experiments using S3I-201. As shown in Figure 6C and 6D, pretreatment with S3I-201 reduced NANOG, SOX2, OCT3/4, Vimentin levels, as well as increasing those of E-cadherin, compared with IL-6 alone. In addition, inhibition of STAT3 suppressed IL-6-induced sphere formation (Fig. 6E, F), suggesting that IL-6 promotes osteosarcoma stemness via activation of STAT3 signaling.

### 7. OPN is involved in IL-6-induced STAT3 pathway activation and enrichment of stemness

Several studies have shown that OPN mediates chemoresistance, recurrence, and migration of osteosarcoma cells 34. Consistent with the findings of Uchibori et al. 35, we also found that IL-6 treatment increased OPN protein levels (P < 0.05) (Fig. 7A, B). To further verify whether OPN can mediate IL-6-induced stemness and STAT3 pathway activation, we pretreated cells with anti-OPN antibody. In agreement with the previous results reported by Choi et al. 36, the expressions levels of NANOG, SOX2, OCT3/4, Vimentin, and a-SMA, as well as the phosphorylation of STAT3, were significantly reduced by treatment with anti-OPN, while levels of E-cadherin were elevated (Fig. 7C, D). The anti-OPN antibody also downregulated IL-6-enhanced sphere formation (Fig. 7E, F). These findings suggest that OPN acts as upstream of IL-6-induced STAT3 activation to promote enrichment of stemness.

### 8. IL-6 promotes osteosarcoma tumor growth *in vivo*

To determine whether IL-6 promotes tumor growth *in vivo*, we used a nude mouse xenograft model. Average tumor volume and weight were measured on day 21 following xenograft injection. As expected, IL-6 treatment increased tumor volume and weight compared with the control group (*P* < 0.05) (Fig. 8A, B). This effect was significantly attenuated by pretreatment with anti-OPN antibodies. Further, we observed an increase in OPN and STAT3 expression levels in osteosarcoma tumor samples in response to IL-6 treatment (Fig. 8C, D). Overall, these data indicate that OPN and the STAT3 pathway participate in IL-6-induced tumorigenesis *in vivo*.

## Discussion

In recent years, the relationships among levels of IL-6 secretion/IL-6-related pathways and chemoresistance, invasion/migration, and acquisition and/or maintenance of stemness features in cancer cells has become a research hotspot. Xiao et al. 18 and Kushlinskii et al. 19 both reported that serum levels of IL-6 were elevated in patients with malignant tumors compared with healthy individuals, and our results support their findings (Table 1). Moreover, our data demonstrate that elevated serum IL-6 levels are correlated with tumor size, tumor, node, metastasis (TNM) stage, and lung metastases, but not with age and sex in patients with osteosarcoma (Table 2). Therefore, we infer that IL-6 may contribute to osteosarcoma progression and acquisition/maintenance of stemness properties.

Lee et al. reported that knockdown of IL-6 leads to retarded tumor growth and lower expression of EMT related markers in CD133^+^ non-small cell lung cancer cells 37. IL-6 can also stimulate the growth, invasion, and migration of prostate cancer cells 38. As shown in Figure 2A, IL-6 significantly elevated proliferation and amplified the clonogenicity of U2OS/MG-63 cells in a time-dependent manner, consistent with the findings of Yu et al. 38. Likewise, migratory/invasive properties are associated with tumor progression. As shown in Figure 3A-G, IL-6 increased the invasiveness of osteosarcoma cells and reduced wound widths in cell migration assays; however, IL-6 did not influence the viability, clonogenicity, or invasion/migration ability of hFOB 1.19 and T98G cells. Moreover, si-IL-6 attenuated the viability, clonogenicity, and invasive/migratory ability of U2OS/MG-63 cells. Overall, these results indicate that IL-6 has specific transforming effects on osteosarcoma cells.

EMT is a crucial biological event involved in cellular transformation, tumorigenesis, and metastasis. In cervical carcinoma, IL-6 induces EMT via STAT3 39, while in lung cancer, IL-6 not only promotes the self-renewal of CD133^+^ CSC-like cells, but also upregulates the expression of EMT-related genes (N-Cadherin, Vimentin, and TWIST), and reduces levels of E-cadherin 40. Similar to previous reports, our findings confirm that IL-6 increases Vimentin and a-SMA levels, and decreases those of E-cadherin, and that these effects can be reversed by treatment with si-IL-6. Numerous studies have proposed improving chemosensitivity by reducing IL-6 production. Hossain et al. found that silencing of IL-6 silencing induces apoptosis and suppresses tumor growth in glioma stem cells 41. Moreover, IL-6 increased chemoresistance to DDR/ADR in U2OS/MG-63 cells, an effect that was reversed by si-IL-6; however, IL-6 had no effect on hFOB 1.19 and T98G cells. Therefore, we conclude that IL-6 exerts a specific effect in maintaining/promoting malignant traits in U2OS/MG-63 cells.

Cortini et al. concluded that co-culturing cells with IL-6 enhances the number of floating spheres, enriched in CSCs, in the osteosarcoma cell population 30. Similarly, IL-6 treatment amplified the number and diameter of U2OS and MG-63-derived spheroids in the current study (Fig. 5A-D). Likewise, tumor-activated mesenchymal stromal cells promote osteosarcoma stemness and migratory potential via IL-6 secretion 42, and si-IL-6 reduces the self-renewal (sphere formation) of the CD133^+^ population among non-small cell lung cancer cells. As shown in Figure 5E-H, IL-6 treatment promoted an increase in the number of CD44- and CD133-positive cells compared with the untreated group at every timepoint (P < 0.05). Wang et al. previously demonstrated that silencing of IL-6 abrogates the expression of OCT4, NANOG, and SOX2, and reduces CSC spheroid diameter among hepatocellular carcinoma CSCs 43. Consistent with those findings, we showed that NANOG, SOX2, and OCT3/4 protein levels were elevated in a time-dependent manner in response to IL-6. Further, si-IL-6 diminished diameters of U2OS/MG-63-derived spheroids and expression of stemness-related markers, validating that IL-6 increases CSC-like phenotypes in U2OS/MG-63 osteosarcoma CSCs.

Increasing evidence suggests that chemotherapy drugs can abolish stem-cell like properties by inhibition of IL-6/STAT3 signaling. Moreover, IL-6 is required for the maintenance of stemness in HER2-positive breast cancer cells, an effect mediated primarily through activation of the STAT3 pathway 44. Our results demonstrated that S3I-201 (a specific STAT3 inhibitor) decreased IL-6-promotion of sphere formation, as well as NANOG, SOX2, and OCT3/4 protein levels, consistent with previous reports.

Overexpression of OPN contributes to the maintenance and enhancement of stemness in various malignancies, including lung, hepatocellular carcinoma, and pancreatic cancer 44-46. Wang et al. showed that overexpression of OPN can mediate IL-6 enhanced cancer stemness and metastasis in hepatocellular carcinoma 43. Furthermore, Choi et al. reported that secretion of OPN led to maintenance of the self-renewal and metastatic capacity of lung CSCs 47. In our study, OPN expression levels were elevated in response to IL-6 (*P* < 0.05) (Fig. 5A, B). Additionally, treatment with an anti-OPN antibody attenuated the effects of IL-6, by decreasing levels of p-STAT3, NANOG, SOX2, and OCT4 (Fig. 5C, D), and reducing sphere formation (Fig. 5E, F). *In vivo*, IL-6 increased the growth of tumors formed from osteosarcoma CSCs, and elevated the levels of OPN and p-STAT3 (*P* < 0.05; Fig. 6) Our data suggest that IL-6 promotes osteosarcoma CSC-like features and chemoresistance by activating STAT3 via OPN *in vitro* and *in vivo*.

Chemoresistance and disease recurrence is an important clinical challenge in patients with osteosarcoma. More work is needed to deepen our knowledge of the role of IL-6 and inflammatory signaling in maintaining osteosarcoma spheroid stemness, and to design more effective anti-CSC therapies. This study provides a framework for the development of novel therapeutic regimens, with the ultimate hope of bringing long-term clinical benefits to patients with osteosarcoma.

## Figures and Tables

**Figure 1:** ** IL-6 expression is correlated with inferior prognosis in patients with osteosarcoma. (A)**Statistical analysis of IL-6 expression levels in osteosarcoma and adjacent non-tumor tissue specimens. **(B)** Association of IL-6 serum expression with clinicopathological traits in patients with osteosarcoma. **(C)** Plasma IL-6 levels were significantly higher in patients with tumor, node, metastasis (TNM) stage III-IV osteosarcoma than in those with stage I-II disease; **(D)** Plasma IL-6 levels were significantly higher in patients with lung metastasis than in those with no lung metastasis.

**Figure 2:** ** The effect of IL-6 on cell proliferation and colony formation. (A)** Normal osteoblastic hFOB 1.19, MG-63/U2OS osteosarcoma, and human glioblastoma T98G cells were treated with or without 10 ng/ml IL-6 for 24, 48, 72 h, and cell viability determined using MTT assays,*p < 0.05 vs. untreated control. **(B)** and **(C)** Representative images of colony formation assays using hFOB 1.19, MG-63/U2OS, and human glioblastoma T98G cells, with or without IL-6 treatment for 24, 48, and 72 h. Data are presented as histograms showing the mean ± SD; *p < 0.05, vs. untreated control. **(D)** and **(E)** Representative colony formation assay plates, with MG-63/U2OS cells treated with or without si-IL-6. Data are presented as histograms showing the mean ± SD; *p < 0.05, vs. si-control group.

**Figure 3:** ** IL-6 accelerates osteosarcoma cell invasion and migration, and promotes EMT. (A-B)** Rate of invasion of hFOB 1.19, U2OS/MG-63, and T98G cells treated with or without IL-6. Right panels, quantitative data. *P < 0.05 vs. corresponding control group. **(C-D)** Rate of migration of hFOB 1.19, U2OS/MG-63 cells, and T98G cells. Right panels, quantitative data. *P < 0.05 vs. corresponding control group. **(E-F)** Levels of E- cadherin, Vimentin, a-SMA, and MMP-2 protein expression. GAPDH was used as a loading control. Results are expressed as means ± SD of three independent experiments; *P < 0.05 vs. corresponding control group. **(G-H)** Transwell analysis was used to detect invasion of U2OS/MG-63 cells, while IL-6 was blocked using si-IL-6. Si-control was used as a loading control. The results are expressed as means ± SD of three independent experiments; *P < 0.05 vs. si-control group. **(I-J )** Rate of migration of U2OS/MG-63 cells with or without si-IL-6 treatment. Right panels, quantitative data. *P < 0.05 vs. si-control group. **(K-L)** E-cadherin, Vimentin, a-SMA, and MMP-2 protein expression levels in MG-63/U2OS cells treated with or without si-IL-6. GAPDH was used as a loading control. Results are expressed as means ± SD of three independent experiments; *P < 0.05 vs. si-control group.

**Figure 4:** ** IL-6 strengthens chemoresistance to DDP/ADR in osteosarcoma cells. (A)** hFOB 1.19, U2OS/MG-63, and T98G cells were pretreated with or without IL-6, then cultured with 0, 0.3, 3, or 30 µg/ml DDP for 48 h. Cell proliferation was determined by MTT assay. *P < 0.05 vs. DDP group alone. **(B)** hFOB 1.19, U2OS/MG-63-CSC, and T98G cells were precultured with or without IL-6, then cultured with 0, 0.06, 0.6, or 6 µg/ml ADR for 48 h. Cell proliferation was determined by MTT assay. *P < 0.05 vs. ADR group alone. **(C)** U2OS/MG-63 cells were precultured with or without si-IL-6, then cultured with 0, 0.3, 3, or 30 µg/ml DDP for 48 h. Cell proliferation was determined by MTT assay. *P < 0.05 vs. DDP + si-control group. **(D)** U2OS/MG-63 cells were precultured with or without si-IL-6, then cultured with 0, 0.06, 0.6, or 6 µg/ml ADR for 48 h. Cell proliferation was determined by MTT assay. *P < 0.05 vs. ADR + si-control group.

**Figure 5:** ** The tumorigenic and self-renewal potential of U2OS- and MG-63-derived spheroids is promoted by IL-6. (A-B)** U2OS/ MG-63/T98G-derived spheroids were isolated and then cultured in the presence or absence of 50 ng/ml IL-6 in serum-free medium. And Morphological observations of hFOB1.19 cells treated with or without IL-6. Each experiment was performed in triplicate. The number and size of spheres formed in U2OS/MG-63/T98G cells were analyzed quantitatively. Data are shown as the means ± SD from three replicates; Scale bar = 100 µm. *P < 0.05 vs. control group. **(C)** The percentage of CD133^+^ cells in U2OS/MG-63-derived spheroids was analyzed by flow cytometry. **(D)** Quantitative analysis of the results shown in C. *P < 0.05 vs. corresponding control group. **(E)** The percentage of CD44^+^ cells in U2OS/ MG-63-derived spheroids was analyzed by flow cytometry. **(F)** Quantitative analysis of the results shown in E. *P < 0.05 vs. corresponding control group alone. **(G-H)** Western blotting was used to estimate the levels of NANOG, SOX2, and OCT3/4 proteins. Right panels, quantitative data. *P < 0.05 vs. control group. **(I-J)** Representative micrographs of spheres formed and the levels of stemness-related genes were analyzed in cells treated with si-IL-6 or si-control. Scale bar, 100 µm. *P < 0.05 vs. si-control group.

**Figure 6:** ** STAT3 signaling pr omotes IL-6-mediated stemness in osteosar coma cells. (A-B)** U2OS and MG-63 cells were treated with or without 50 ng/ml IL-6 for 24, 48, and 72 h. Activation of STAT3 was assessed by western blotting. GAPDH was used as a loading control. Results are expressed as means ± SD (n = 3 independent experiments). *P < 0.05 vs. control group. **(C-D)** U2OS- and MG-63-derived CSCs were pretreated with 10 μM of S3I-201 for 1 h in the presence or absence of IL-6. Western blot analysis was used to determine the protein levels of NANOG, SOX2, OCT3/4, p-STAT3, STAT3, Vimentin, a-SMA, and E-cadherin. GAPDH was used as a loading control. Results are expressed as means ± SD (n = 3 independent experiments). *P < 0.05 vs. control group; &*P* < 0.05 vs. IL-6 group. **(E-F)** Osteosarcoma CSCs were treated with or without IL-6 in the absence or presence of S3I-201. After treatment, cells were assayed for sphere formation. *P < 0.05 vs. control group; & *P* < 0.05 vs. S3I-201 group. Scale bar, 50 μm. All data are representative of three independent experiments.

**Figure 7:** ** OPN is involved in IL-6-induced STAT3 pathway activation and stemness enrichment. (A-B)** OPN protein levels were measured by western blotting. Right panels, quantitative data. *P < 0.05 vs. control group. **(C-D)** NANOG, OCT4, SOX2, and p-STAT3 levels were determined by western blot. Results are expressed as means ± SD of three independent experiments; *P < 0.05 vs. control group; &*P* < 0.05 vs. IL-6 group. **(E-F)** Single-cell suspensions from primary U2OS and MG-63 cells were seeded at 5 × 10^4^/well in 96-well plates; sphere formation occurred after 7 d. Sphere size and cell number were quantified using microscopy. *P < 0.05 vs. control group; &*P* < 0.05 vs. IL-6 group.

**Figure 8:** ** IL-6 augments the tumorigenic properties of osteosarcoma spheroids *in vivo*. (A)** Representative images of primary osteosarcoma tumors. Control or IL-6-treated osteosarcoma cells were injected subcutaneously into nude mice. *P < 0.05 vs. control group. **(B)** Tumor growth curves. Tumor size and weight were measured after excision from mice (n = 5). *P < 0.05 vs. control group. **(C-D)** OPN and p-STAT3 levels in tumor tissues were measured by western blotting. Right panels, quantitative data. *P < 0.05 vs. control group.

**Table 1:** Statistical analysis of IL-6 expression in osteosarcoma and control groups

Groups	n	IL-6 expressions	P values
Control	50	93.26±50.62	P<0.05
Osteosarcoma	54	271.92±90.81	

**Table 2:** The relationship between serum of IL-6 and pathological characteristics in osteosarcoma patients (pg/ml)

Characteristic	n (%)	IL-6 expression	P values
**Gender**			
Male	36	278.62±60.37	0.325
Female	18	267.87± 30.60	
**Age(years)**			
<20	31	276.72±60.37	0.187
**≧**20	23	268.79±34.74	
**Tumor size**			
≤5	20	289.36±40.36	0.376
>5	34	272.67±35.80	
**TNM stages**			
I-II	30	251.92±30.31	0.023*
III-IV	24	311.23±20.81	
**Lung metastasis**			
No	33	249.88±40.82	0.017*
Yes	21	303.93±29.29	

*P<0.05
